The article "Mediating the performance of social organizations in context of social and organizational innovations in China" was retracted in 2024. Reasons: concerns about the data; concerns about the results or conclusions; concerns about the peer review; concerns about the authorship.

# Mediating the performance of social organizations in context of social and organizational innovations in China

**DOI:** 10.1371/journal.pone.0281720

**Published:** 2023-03-24

**Authors:** Tang Tao, Ghulam Rasool Madni, Iftikhar Yasin

**Affiliations:** 1 Institute of Xi Jinping Thought on Socialism with Chinese Characteristics for a New Era, Peking University, Beijing, China; 2 Department of Economics, Division of Management and Administrative Science, University of Education, Lahore, Pakistan; 3 Department of Economics, The University of Lahore, Lahore, Pakistan; University of Salento, ITALY

## Abstract

Social and organizational innovations are one of the most effective ways to gain social collaboration for effective, rapid, and coordinated interventions. An analysis of the relationship among organizational performance (OP), social innovations (SI) and organizational innovation (OI) in social organizations (SOs) is little discussed in the literature and much less with main component analysis. This paper is an effort to provide some empirical evidences about social and organizational innovations that social organizations in China have implemented to address the social issues of the society. A survey of Chinese SO’s is conducted during beginning two months of 2022 in provinces of Jiangsu, Guangdong and Zhejiang to attain the statistics and assessing the insights of the executives of the SOs participating in this study with respect to organizational performance, social and organizational innovations. The technique used to select the sample is a non-probabilistic sampling and multiple linear regression model is applied to determine the partial impact of organizational innovations and social innovations on the organizational performance. The grouping of the variables is carried out through main components analysis. The empirical findings of the study highlight that Chinese SOs are innovative because they adopt management strategies to address the social issues associated with their institutional mission. There are four groups of derived components from organizational and social innovations based on the empirical evidence: SO’s innovative activities to modify the environment; inside innovative measures to enhance SO’s performance; innovative activities of SO’s to enhance their relationships with outside actors; innovative measures to improve the management of SOs related to their mission and institutional projects. The findings of this study offer an efficient solution to government and policy makers for involving SOs in terms of planning of social development in China. The social and organizational innovations are very necessary to overcome the social issues so government should encourage the establishment and sustainability of social organizations.

The article "Mediating the performance of social organizations in context of social and organizational innovations in China" was retracted in 2024. Reasons: concerns about the data; concerns about the results or conclusions; concerns about the peer review; concerns about the authorship.

## 1. Introduction

The invention and execution of novel ideas (processes, services, and products,) to meet societal demands are known as social innovations [1]. It is worth noting that social innovations (SIs) are not limited to SOs that work to solve social issues but it is a kind that responds to societal requirements in corporate organizations in exchange for the social advantages they gain [2,3]. It should not be utilized as a strategy by organizations engaged in this activity to increase economic benefits [4]. According to Mumford [5], SI is the implementation and development of innovative ideas for how individuals might organize social interactions or interpersonal activities to achieve some common goals with social benefits while Levesque [6] is of view that it is a process that contributes to novel solutions to intractable societal issues.

Organizational Innovation (OI) is defined by [7] as advances in inside interactions in an organization, like collaborations among different units, as well as affiliation and engagement among various interest groups and their networks (other research laboratories, assistance services, companies, etc.). The study [8] sees it as a fundamental shift in organizational management, procedures, routines, strategic orientation, and structure. Innovation entails learning procedures in organizations that foster abilities, teamwork knowledge, adaptation to environment, and facilitating competitiveness [9].

Although there is no widely agreed definition, most researchers perceive that organizational performance is the assessment of variety of factors, including the evaluations of process and the outcomes of various organizational actions [10,11]. In this regard, SOs confront three distinct obstacles in terms of performance results: meeting stakeholder expectations, meeting internal needs to optimize effect, and utilizing results for learning and improvement [9].

The importance of SOs in developing countries is growing, owing to the need for innovative methods in a variety of uncertain, diverse, and complicated social environment. These tactics should assure SOs long-term viability in association with improving solutions to societal problems [12]. To develop, execute, and offer excellent services to their consumers, SOs require innovative tactics, as well as to deal with increasing competitiveness for funds, the complications of societal problems resulting from evolving issues, and donors who demand higher levels of transparency and more efficient management [13,14]. Furthermore, these organizations are also contributing to create large number of jobs and volunteers in developing countries. Furthermore, it is critical to emphasize that social organizations are critical in developing economies. SOs demand more incentives to improve their efficacy and efficiency, as well as their overall competitiveness [15,16]. Various research studies have supported this viewpoint, demonstrating a direct link between SO innovation and performance efficiency [16–21].

The article "Mediating the performance of social organizations in context of social and organizational innovations in China" was retracted in 2024. Reasons: concerns about the data; concerns about the results or conclusions; concerns about the peer review; concerns about the authorship.

Since the year 2000, social innovations have been a widespread concept in China. “Social Innovation Management" is a significant driver of innovations in public sector, while activities related to social entrepreneurship continue to inspire numerous innovative projects in the private sector. The Chinese government began taking steps in 2010 to encourage SOs to start providing social services because the relationship between the Chinese government and SOs had previously been marked by political conflict. This move drew considerable attention from both domestic and foreign observers. In contrast, it appeared that the government was not only willing to pay SOs, but was also willing to provide assistance to help SOs to expand their capacity and provide additional social services. SOs expanded in number tremendously as a result of this governmental incentives. By the end of 2015, China had over 600000 SOs in function, employing 7.35 million people and 4696 charity foundations. This shift in the interaction between the state and the private sector has had a major effect on development of China’s social policy. It has affected not only the bodies that offer social services, but also the content of those services and the decision-making procedures that go along with them. SOs have now become an important aspect of Chinese social life. China altered its industrialization policy from investment based production and labor intensive industry to innovation-oriented growth in the early days of economic reform in the late 1990s, following high growth that headed to new sorts of development. The government document "Decision on Accelerating the Progress of Science and Technology," published in 1995, is an example of state’s regulations towards technological innovations, strongly stressed on technological and managerial innovations. In addition, this policy emphasized the importance of social innovations in social and commercial sectors. After mid-2000s, innovative initiatives in the social sector were primarily focused in two policy areas: social management at the community and local levels, and service area. The government promoted a business sector policy of mass entrepreneurship and innovation, advocating for adoption of development through innovations as a national strategy. The importance of social innovations as a national development guide is also highlighted.

The article "Mediating the performance of social organizations in context of social and organizational innovations in China" was retracted in 2024. Reasons: concerns about the data; concerns about the results or conclusions; concerns about the peer review; concerns about the authorship.

Many firms have pushed and exercised the standards of corporate social responsibility (CSR) when it comes to social innovations in workplace and improved the efficiency of human resource management since the mid-2000s. Furthermore, following the 2008 Wenchuan Earthquake in China’s Sichuan province, the private charity sector exploded. The creation of charitable platforms improved the transparency of donations, encouraging private companies to participate actively in charitable operations. Social organizations (SOs) are still the private sector’s innovative agents for creating welfare resources. Local governments have also been given a substantial amount of public funding to carry out social programs and provision of services by supporting their financial ability. Fig 1 depicts the number of social organizations in China with the passage of time.

**Fig 1:** Source: China Philanthropy Times (20-01-2021).

According to the China Social Organization Network, China had 320,000 social organizations in 2012. The number increased to 390,000 in 2013 and has continued to rise. China’s total number of registered social organizations was 890,000 by 2020. By 2021, China has registered 900,914 social organizations in compliance with the law and more than 1 million social organizations are expected to operate in the country by the end of 2022. Jiangsu, Guangdong, and Zhejiang are the three provinces with the most registered social organizations. Up until now, there are 11 provinces; Anhui, Fujian, Guangdong, Guangxi, Henan, Hubei, Hunan, Jiangsu, Shandong, Sichuan, Zhejiang—with more than 30,000 social organizations. With about 98,000 social organizations and the potential to approach 100,000 in the near future, Jiangsu ranks top among the 11 provinces. With over 70,000 social organizations in each region, Guangdong and Zhejiang Provinces come in second and third, respectively. Shandong Province, which has more than 60,000 social organizations, followed Guangdong and Zhejiang Province in having the most. The remaining provinces each have fewer than 50,000 social organizations. In the four central-administered municipalities, Chongqing has the largest number of social organization registrations (18,000), followed by Shanghai (17,000), Beijing (14,000) and (6,500) in Tianjin (China Philanthropy Times, 20-01-2021).

More research on the relationship between performance of SOs and innovations is clearly needed, especially with reference to emerging economies [16,18,22]. Furthermore, the present findings are inconclusive. The study [23] point out that stakeholders evaluate the SOs from a variety of perspectives. Many aspects of SI and OI involve change in work formats that are not always directly realized by concerned groups, resulting in a wide range of findings from different studies. The SOs in the emerging economies have still lacking a systematic measurement culture [18]. This research aims to discover the social and organizational innovations used by SOs in the last five years, focusing on the innovations that have had the most impact on these organizations. Furthermore, this research aims to examine the OIs and SIs made by Chinese SOs in terms of their relationship to their management and ways to address their mission regarding social issues. It is intention of the study to contribute in empirical evidence for understanding the relation among organizational performance, organizational and social innovations by SOs in China. This study is a pioneer study investigating the relationship among social and organizational innovations with organizational performance of social organizations in China. For the purpose, primary data is collected through questionnaires. Then descriptive analysis, multiple regression analysis and main component analysis are carried out to devise some fruitful conclusions based on collected data. It is found that social organizations are important to tackle the social issues of China. Furthermore, social and organizational innovations are necessary for sustainability of these organizations. If suitable working environment persists then organizations are in better position to innovate.

The article "Mediating the performance of social organizations in context of social and organizational innovations in China" was retracted in 2024. Reasons: concerns about the data; concerns about the results or conclusions; concerns about the peer review; concerns about the authorship.

## 2. Methodology

The SOs in three provinces of China (Jiangsu, Guangdong, and Zhejiang) are the source of information for this study. The aims and methods of the study were explained in invitation letters sent to 480 organizations. The consent was given by 192 organizations to participate in the survey while 163 organizations accomplished the survey. The “Ethical Review Committee” of the University of Education approved the study and its format. The sample of social organizations is diversified by including the charitable SOs (provision of housing, clothing or medicine; distribution of food etc.), business foundations (provision of schools, shelters, housing etc.), social associations (for the marginalized groups, pensioners, disabled, etc.), community SOs (gender, educational, religious, etc.), defense or protection (of immigrants, women, children, human rights, animals, environment, etc.). Those organizations were included in the sample who have at least 5 years of operations at the time of survey (surveyed organizations have 10 years of operation on average) and have a pay roll of 12 full time workers (the average workers in sample organizations were 35). Among the sample organizations, 18% are international while 82% are national social organizations.

The article "Mediating the performance of social organizations in context of social and organizational innovations in China" was retracted in 2024. Reasons: concerns about the data; concerns about the results or conclusions; concerns about the peer review; concerns about the authorship.

Based on research objectives and earlier literature, the authors developed a survey format following [23] to analyze the relationship among organizational performance, organizational and social innovations. Before sending the questionnaire, a written consent form was sent to participants. The participants who filled the consent form in written and showed their willingness to participate, were given the questionnaire. The participants were free to leave the survey at any stage. The questionnaire has three parts: social innovations, containing 10 main items determined through [1,24–27]; organizational innovation, based on 20 items determined through [19,28–30]; and organizational performance consisting of 8 items determined through [31,32]. Each item in the section has relevance with that section as highlighted in the earlier studies. The theoretical relationship of each item is developed through the definition of each part.

These 3 sections are analyzed on Likert scale ranging from one to five where: 1 = strongly disagree, 2 = partially disagree, 3 = indifferent, 4 = partially agree while 5 = strongly agree. The questionnaire is pilot tested by twelve executives of sampled social organizations. With the suggestions and proposals of these executives, deficiencies were recognized and then questionnaire is used to gain the data of SO’s. The researchers visited the managers of the participating social organizations in person at their work sites during the January and February 2022.

Fisher F test is used to determine the partial impact of the independent variables (organizational and social innovations) on the dependent variable (organizational performance). The statistical tests are also applied to check the validity of regression assumptions; White’s Test for homoscedasticity; Durbin Watson (DW) test to determine the non-correlation of error term while the Shapiro Wilks test to find the normality of error term.

## 3. Results

The findings of the study are presented on three levels: a) descriptive analysis; to determine the SI, OI, and OP, b) multiple regression models to illustrate the effect of OI and SI on the performance of the SOs, explaining the behavior of each variable c) main component analysis (MCA) to categorize the groups of OI and SI actions that participate in changes, responsible for performances of these organizations.

### 3.1. Descriptive analysis

Generally, executives of the organizations mentioned that their organizations have engaged in a variety of innovative activities over the last three years (SI received an average score of 4.11/5.0, and OI received an average score of 4.04/5.0), and that OP scored an average of 4.11/5.0). These findings suggest that SOs value innovation as one of their objectives for achieving their organizational goals. It is noteworthy that the participants of this study showed a positive attitude towards innovation which demonstrates that these organizations are concerned about the demands and challenges of societal issues confronting the developing countries. Moreover, these organizations are aware about the complexity of these problems and working to combat them.

The article "Mediating the performance of social organizations in context of social and organizational innovations in China" was retracted in 2024. Reasons: concerns about the data; concerns about the results or conclusions; concerns about the peer review; concerns about the authorship.

These findings suggest that SOs’ willingness to engage in both OI and SI is might be due to prevailing competition in China among social organizations to acquire funding from the donors and government. These donors want to finance those projects who have transparency and efficiency so resource may be used optimally. It is also evident from the results that various actors in China are requiring greater professionalism in the management of SOs for resource allocation in order to work with unprivileged groups.

The averages of each item included in the sections of SI, OI, and are shown in Table 1. For Social Innovation, a maximum average value was attained in "Development in the ability of SO to recognize, integrate, transform, and use of external information in order to solve societal issues related with goal of SO" with 4.38, and the lowest value was 3.94 for “Several members of the SO have recognized societal needs that are relevant to the organization’s mission”. Regarding the items of Organizational Innovation, the highest average is recorded in the item, "Positive adaptability to changes in the environment" with score of 4.44 and the lowest average value (3.68) is for "There is change in human resource management" (Table 2). Finally, for Organizational Performance, the highest value of 4.33 is for “There is improvement in relationship with users”. The lowest was “Diverse funding sources are expanded for progress” with 3.55 (Table 3).

**Table 1:** Average percentage in the items of social innovations.

Item	Social Innovations	Average
1	Development in the ability of SO to recognize, integrate, transform, and use of external information in order to solve societal issues related with goal of SO	4.38
2	Innovative methods and processes have been implemented to deliver services	4.24
3	Working in conjunction with external actors to exchange knowledge and information to meet the mission of SO	4.21
4	Several members of the SO have recognized societal needs that are relevant to the organization’s mission	3.94
5	For the growth of organization’s social projects, there are a variety of sources (users, seminars, experts and academic reports by institutions, etc.) exist	4.11
6	The collaboration among partners for the progress of social projects in line with institutional mission is diverse	4.01
7	Initiatives encouraging users to work together in addressing the problems have been encouraged	4.22
8	There are several modes of social actions	3.98
9	The social projects have produced a wide range of results in terms of sectoral effect	3.99
10	Projects are resulted in the creation of new organizational infrastructure	4.01
	**Average Social Innovations**	4.11

The article "Mediating the performance of social organizations in context of social and organizational innovations in China" was retracted in 2024. Reasons: concerns about the data; concerns about the results or conclusions; concerns about the peer review; concerns about the authorship.

**Table 2:** Average percentage in the items of organizational innovations.

Item	Organizational Innovations	Average
11	Positive adaptability to changes in the environment	4.44
12	Changes in the environment are quickly absorbed by management	4.01
13	Organizational performance has improved as a result of improvements in management style	4.11
14	Managers have implemented improvements that enable employees to be more productive	4.27
15	To achieve better performance, managers have encouraged their workers to change their attitudes	4.31
16	Modifications in work processes lead to the creation of new and improved services	4.08
17	The adoption of new technology to boost the performance of employees and improving their services have been encouraged	3.99
18	Human resource create their own methods of working	4.02
19	The staff positions have altered as a result of the SOs’ situation	3.89
20	The decisions of management are made on the basis of changing demands	3.92
21	There is change in human resource management	3.68
22	Ways of interaction with customers are modified	4.12
23	There is change in relationship with donors	3.95
24	There is change in relationship with community	4.22
25	Personnel initiatives has been encouraged by management in order to find new sources of funding	4.12
26	Cooperation between SOs and other private or private bodies has been encouraged in order to improve services	3.86
27	There is change in organizational structure in response to changes in the external and internal environment	4.13
28	There is change in job responsibilities	3.84
29	Training activities are repeated on regular basis to improve the performance of workers	4.14
30	The sharing of knowledge, expertise, ideas, and related information has been encouraged among members of the organization to strengthen the organization’s activities	3.74
	**Average Organizational Innovation**	4.04

**Table 3:** Average percentage in the items of organizational performance.

Item	Organizational Performance	Average
31	Organizational culture of social organization has been developed	4.11
32	There is improvement in relationship with users	4.33
33	The effectiveness of social organization has upgraded in order to improve their objectives and mission	3.97
34	Diverse funding sources are expanded for progress	3.55
35	Perceptions about the requirements of users have been improved	4.13
36	Associated team work between community agents and SO	4.21
37	Efficiency in resource utilization to meet objectives has been improved.	4.35
38	Presented findings have been used to achieve the institutional objective	4.27
	**Average Organizational Performance**	4.11

The article "Mediating the performance of social organizations in context of social and organizational innovations in China" was retracted in 2024. Reasons: concerns about the data; concerns about the results or conclusions; concerns about the peer review; concerns about the authorship.

### 3.2. Multiple Regression Analysis (MCA)

To analyze the effect of different items of SI and OI on performance of SOs, a multiple linear regression model is used to determine the trend and relationship among 7 dependent variables (performance items) relying on 30 items relevant to independent variables (innovative actions). Multiple regression analysis considers all potential important factors in a model and provides more precise and accurate relationship among each individual items of the model along with its outcomes. Simple linear regression may be applied but it is efficient in case of univariate analysis and may provide misleading results if there is multivariate analysis. If outcome of interest is suspected to be associated with more than one predictors, then MCA is more appropriate. Moreover, a model having simultaneous multiple predictor variables then MCA provides efficient empirical results.

In Table 4, it is shown that Fisher F test is applied on each multiple linear regression model and found 95% confidence level determined by p-value. It provides strong evidence to believe that independent variables explain the variability of the dependent variable. For example, the item 5 which is performance of SOs (dependent variable), is relevant to enhance the real knowledge of users of SO. In addition, the linear regression model consisting of thirty items is linked with SI and OI explaining 79.4% (R^2^) of the performance variability.

**Table 4:** Activities of OI and SI explaining percentage variability of organizational performance.

Item	Aspects of the Organizational Performance	R^2^	df	F	P-Value
1	Organizational culture of social organization has been developed	0.718	30	3.113	0.002
2	There is improvement in relationship with customers	0.827	30	4.314	0.001
3	The efficiency of social organization has upgraded in order to improve their objectives and mission	0.743	30	2.982	0.005
4	Diverse funding sources are expanded for progress	0.751	30	2.636	0.003
5	Perceptions about the requirements of users have been improved	0.794	30	5.172	0.001
6	Associated team work between community agents and SO	0.816	30	4.171	0.002
7	Efficiency in resource utilization to meet objectives has been improved.	0.811	30	3.537	0.004
8	Presented findings have been used to achieve the institutional objective	0.724	30	3.462	0.003

Table 5 shows the factors having a greater relative impact on the dependent variables, using standardized regression coefficients as a criterion.

The article "Mediating the performance of social organizations in context of social and organizational innovations in China" was retracted in 2024. Reasons: concerns about the data; concerns about the results or conclusions; concerns about the peer review; concerns about the authorship.

**Table 5:** OI and SI activities explaining the main aspects of OP.

Dependent Variable (SO performance)	Standardized ‘d’ regression coefficient	Innovation’s aspect with greater relative influence
(1) Organization’s cultural improvement	0.128	10. Projects are resulted in the creation of new organizational infrastructure
	0.132	8. There are several modes of social actions
	0.114	18. Human resource create their own methods of working
	0.081	28. There is change in job responsibilities
	0.084	23. There is change in relationship with donors
	0.069	26. Cooperation between SOs and other private or private bodies has been encouraged in order to improve services
(2) Improvements in relationship with users	0.369	10. Projects are resulted in the creation of new organizational infrastructure
	0.221	8. There are several modes of social actions
	0.134	13. Organizational performance has improved as a result of improvements in management style
	0.089	2. Innovative methods and processes have been implemented to deliver services
	0.079	21. There is change in human resource management
(3) Improvements in developing the mission of SOs	0.361	10. New Organizational infrastructure is created through projects.
	0.188	8. There are several modes of social actions
	0.159	26. Collaborated actions among SOs, private and public entities have been promoted to improve the service.
	0.146	23. Sponsor’s relationships have changed.
	0.085	18. Development of work approaches by Human resources.
(4) Diversity in sources of project financing	0.872	10. Projects are resulted in the creation of new organizational infrastructure
	0.141	23. There is change in relationship with donors
	0.173	8. There are different social intervention modes.
	0.149	26. Cooperation between SOs and other private or private bodies has been encouraged in order to improve services
	0.151	3. Working in conjunction with external actors to exchange knowledge and information to meet the mission of SO
(5) Improved knowledge	0.131	12. Changes in the environment are quickly absorbed by management
	0.157	16. Modifications in work processes lead to the creation of new and improved services
	-0.268	19. The staff positions have altered as a result of the SOs’ situation
	0.241	24. There is change in relationship with community
	0.282	1. Development in the ability of SO to recognize, integrate, transform, and use of external information in order to solve societal issues related with goal of SO
(6) Joint team work between community agents and SOs	0.136	23. There is change in relationship with donors
	0.131	26. Cooperation between SOs and other private or private bodies has been encouraged in order to improve services
	0.182	29. Training activities are repeated on regular basis to improve the performance of workers
	0.173	2. Innovative methods and processes have been implemented to deliver services
	0.114	3. Working in conjunction with external actors to exchange knowledge and information to meet the mission of SO
(7) Efficient usage of resources	0.179	11. Positive adaptability to changes in the environment
	0.143	13. Organizational performance has improved as a result of improvements in management style
	0.174	21. There is change in human resource management
	0.251	4. Several members of the SO have recognized societal needs that are relevant to the organization’s mission
	0.232	14. Managers have implemented improvements that enable employees to be more productive

This study identified the actions of SI and OI in Chinese SOs linked with OP such as: “Improvement in Organizational Culture, Improvement in Relations with Users, The Increase in the Effectiveness of SOs in Carrying out their Mission, The Diversity of Sources of Financing for Institutional Projects, Better Understanding of User Needs,Consolidation of Teamwork between the SO and Community Agents, Greater Efficiency in the Use of the SO’s Resources for the Development of its Mission and, The Best Results in Achieving the SOs Objectives.”

The article "Mediating the performance of social organizations in context of social and organizational innovations in China" was retracted in 2024. Reasons: concerns about the data; concerns about the results or conclusions; concerns about the peer review; concerns about the authorship.

### 3.3. Main components analysis

With the aforementioned data collection that makes social and organizational innovations in Chinese social organizations, main component analysis is used to decrease the data through correlation analysis. Main component analysis (MCA) has advantage to provide more accurate results in spite of low accuracy of model. It has the ability to reduce the data noise and to produce uncorrelated and independent characteristics of the observations. MCA has more efficiency to transform the high dimensional data to low dimensional data. It has the ability to remove the correlated features and reduces overfitting of the model. It keeps the maximum amount of information in data of the model. The obtained p-value (shown in Table 6) and value of Barlett Sphericity test (0.878) indicate the rejection of null hypothesis; thus, there is significant correlation and relationship among the innovation variables, and main component analysis is appropriate for further analysis.

**Table 6:** Appropriateness for applying the main component analysis.

Kaiser-Meyer-Olkin Measure of Sampling Adequacy		0.878
Barlett’s Sphericity test	Approx. Chi-squared	2,271.516
	Degrees of freedom	703
	P-value	0.003

Table 7 demonstrates the changes in the overall variance as the number of components increase. The aspects of innovations or variables are grouped into four components explaining about 83 percent of variability of total sampled data. The squared cosines of each variable are used to allocate each item to one of the four components, resulting in the formation of the components given in Table 8.

The article "Mediating the performance of social organizations in context of social and organizational innovations in China" was retracted in 2024. Reasons: concerns about the data; concerns about the results or conclusions; concerns about the peer review; concerns about the authorship.

**Table 7:** Total variance explained by the factors.

Number of components	Initial Eigenvalues			Sum of Squared Loading		
	Total	% Variance	% Accumulated	Total	% Variance	% Accumulated
1	11.743	47.266	39.286	11.743	47.266	36.299
2	3.002	14.725	49.152	3.002	14.725	59.152
3	1.613	11.874	70.602	1.613	11.874	68.618
4	1.476	9.259	51.884	1.476	9.259	79.843
5	1.238	5.384	56.284	1.238	5.384	81.571
6	1.079	2.513	83.271	1.079	2.513	84.226
7	0.880	1.100	84.537			
…	…	…	…			
30	0.212	0.458	100.000			

**Table 8:** Grouping of variables based on square cosines.

Description of the factor	Performance Indicators	Average
1. SO’s adaptation to environment	4. Several members of the SO have recognized societal needs that are relevant to the organization’s mission	3.68
	11. Positive adaptability to changes in the environment	4.35
	12. Changes in the environment are quickly absorbed by management	3.96
	14. Managers have implemented improvements that enable employees to be more productive	4.12
	15. To achieve better performance, managers have encouraged their workers to change their attitudes	4.05
	20. The decisions of management are made on the basis of changing demands	4.13
	27. There is change in job responsibilities	3.74
	28. Training activities are repeated on regular basis to improve the performance of workers	3.43
	30. The sharing of knowledge, expertise, ideas, and related information has been encouraged among members of the organization to strengthen the organization’s activities	4.25
2. Changes in management of SO	1. Development in the ability of SO to recognize, integrate, transform, and use of external information in order to solve societal issues related with goal of SO	4.23
	2. Innovative methods and processes have been implemented to deliver services	3.76
	16. Modifications in work processes lead to the creation of new and improved services	4.25
	17. The adoption of new technology to boost the performance of employees and improving their services have been encouraged	4.03
	18. Human resource create their own methods of working	3.92
	19. The staff positions have altered as a result of the SOs’ situation	4.00
	21. There is change in human resource management	3.80
	29. Training activities are repeated on regular basis to improve the performance of workers	3.81
3. Consolidation with external agents	3. Working in conjunction with external actors to exchange knowledge and information to meet the mission of SO	4.18
	5. For the growth of organization’s social projects, there are a variety of sources (users, seminars, experts and academic reports by institutions, etc.) exist	3.97
	6. The collaboration among partners for the progress of social projects in line with institutional mission is diverse	3.96
	7. Initiatives encouraging users to work together in addressing the problems have been encouraged	4.31
	12. Changes in the environment are quickly absorbed by management	4.38
	23. There is change in relationship with donors	4.06
	24. There is change in relationship with community	4.01
	26. Cooperation between SOs and other private or private bodies has been encouraged in order to improve services	4.03
4. Management of social projects	8. There are several modes of social actions	4.03
	9. The social projects have produced a wide range of results in terms of sectoral effect	4.29
	10. Projects are resulted in the creation of new organizational infrastructure	3.89
	22. Ways of interaction with customers are modified	4.07
	25. Personnel initiatives has been encouraged by management in order to find new sources of funding	3.84

It’s vital to note that the initial Eigenvalues represent the results of 30 initial items, whereas the sum of squared loading represent the results when working with 6 components as shown in Table 7. However, we focused the empirical findings of first four components, which better described the variance of data. After analyzing the squared cosines of variables included in the main components analysis, they are classified into four components as highlighted in Table 5. Each factor’s variables are correlated, and majority of them pertain to a common theme that permits each component to assign a name. As a result, component 1 includes innovation actions of social organizations regarding adaptation to environment. Component 2 combines the factors linked with internal innovations of social organizations targeted to improve their performance, with a focus on human management. Component 3 incorporates the variables entailing the innovation actions of SOs to strengthen their relationships with external agent such as private, public, and users’ entities. Finally, Component 4 combines the variables relevant to innovation initiatives aiming at strengthening the management of social programs linked with SOs’ mission and management of institutional project.

The article "Mediating the performance of social organizations in context of social and organizational innovations in China" was retracted in 2024. Reasons: concerns about the data; concerns about the results or conclusions; concerns about the peer review; concerns about the authorship.

Table 8 demonstrates that component 1 contains 7 items and has the greatest relevance to the adaptation to the environment and evidenced as “Positive adaptability to changes in the environment” (4.35); “The sharing of knowledge, expertise, ideas, and related information has been encouraged among members of the organization to strengthen the organization’s activities” (4.25); “The decisions of management are made on the basis of changing demands” (4.13), and the items of less relevance are “Training activities are repeated on regular basis to improve the performance of workers” (3.43) and in “There is change in job responsibilities” (3.74). The component 2 has eight items and most relevant to internal changes in the administration is the “Modifications in work processes lead to the creation of new and improved services” (4.25), and “Development in the ability of SO to recognize, integrate, transform, and use of external information in order to solve societal issues related with goal of SO” (4.23), and the least relevant is the “There is change in human resource management” (3.80). The component 3 has eight items and most related to integration with external agents is “Changes in the environment are quickly absorbed by management” (4.38), and “Initiatives encouraging users to work together in addressing the problems have been encouraged” (4.31); and the least relevant is the “The collaboration among partners for the progress of social projects in line with institutional mission is diverse” (3.96). The component 4 has seven items and most related to management of social intervention and projects is “Fostering the link with external agents for the exchange of information”, and “The social projects have produced a wide range of results in terms of sectoral effect” (4.29); the least relevant is “Personnel initiatives has been encouraged by management in order to find new sources of funding” (3.84).

## 4. Discussion and conclusion

This research paper is intended to analyze the relationships among social innovations, organizational Innovation, and organizational performance in social organizations of China. The earlier literature on the topic highlights that there is very short literature in context of emerging and developing economies. Moreover, the existing literature has inconclusive findings. The role of social organizations in solving social problems is inevitable now days so importance of the exploration of the topic as increased manifold. The findings of this study contribute in the literature of social organizations in the following ways:

Firstly, empirical findings of the study highlight that social organizations in China are innovative organizations which use management approaches to achieve their goals. Changes in management techniques, work methods, organizational structure, connections with donors, and the deployment of new tactics for collaborative work with private and public organizations are all instances of purposive strategies. These findings are consistent with [2,33], who found that because SOs confront a highly complicated, competitive, uncertain, and globally connected environment along with growing scarcity of resources, the outcome is some significant improvements in innovations stemmed from interactions of donors and funders. However, [34–36] have contrasting findings and provide evidences that SOs even from developing countries place little attention to innovations as a survival strategy, owing to measures of their resistance to change and low tolerance for risk. The Chinese SOs in this research, have been distinguished for their willingness to address the social concerned to their institutional mission. The innovative strategies used by these organizations to determine the requirements of donors is an illustrative example. In addition, searching additional resources for social programs of SOs, the utilization of new options to tackle social problems, the diversity of partners for project development, and management techniques that involve working in teams with donors are few examples.

The article "Mediating the performance of social organizations in context of social and organizational innovations in China" was retracted in 2024. Reasons: concerns about the data; concerns about the results or conclusions; concerns about the peer review; concerns about the authorship.

These findings enable us for a well understanding of social innovations in SOs. According to [2,37,38], there is little focus in the research on the dynamics and nature of innovations carried out by SOs, especially when these innovations contribute in solving the societal issues because the outcomes of earlier studies on the subject topic needs to be concluded [39,40]. Researching the social innovations by SOs in context of socioeconomic circumstances of China is critical since the country has a big population. Furthermore, owing to lack of quality in daily life, a huge Chinese population face difficulty to meet fundamental demands. According to [27,41], SOs require new approaches, plans, processes, and initiatives for collaboration among government agencies and donors in order to contribute by employing innovative strategies to solve the social problems.

The second evidence shows that SI and OI by social organizations of China significantly explain each aspect linked with organizational performance like 1) improvement of organizational culture; 2) improvement in relations with donors; 3) improvement in efficiency of SOs’ in pursuing their institutional mission; 4) diversity of sources of funding for organizational projects; 5) best knowledge about needs of users; 6) improvement in efficiency regarding utilization of resources to meet the mission of organizations; 7) consolidated team work between community agents and social organizations. These findings are in line with evidences of [16,22,26,42], each of whom conclude that there is a positive relation between innovation actions and performances of SOs.

The article "Mediating the performance of social organizations in context of social and organizational innovations in China" was retracted in 2024. Reasons: concerns about the data; concerns about the results or conclusions; concerns about the peer review; concerns about the authorship.

The third one is based on evidence that the main components arising from SI and OI by social organizations are divided into four categories: the first one relates to adaptation of social organization to its environment; the second group is about internal innovations of social organizations that improves their management; third group includes innovative actions improving the relationship with external agents like donors, public and private agencies; while the fourth group is about the innovative efforts targeted to enhance the management of social organizations related with management of institutional projects and mission of SOs.

The recognition of key components of OI and SI that affect the performances of social organizations is very important due to their serving as a reference guide of SOs. This study also contributes to answer the concerns of [35] who explain that in spite of importance of innovations to improve the organizational performance, many social organizations are resist the innovations for economic gains. This resistance occurs due to unawareness of managers about the importance of innovations for their organizations. Furthermore, because social organizations in developing countries are typically highly formal, centralized in decision-making, and standardized in their procedures, they suffer from a lack of flexibility in the orientation of their users, a lack of commitment to their mission, and strict control by political and regulatory institutions [36]. The findings of [34] describe that resistance in these organizations occur due to failure of development of social skills necessary for social innovations.

Since the mid-2010s, China has encouraged social innovations as a national development strategy. For social innovations, new concepts, organizational behavior models, agendas, and policy initiatives have been tested. These advances foster an environment that encourages social innovations in general. "Coordination, ecology, openness, and sharedness" are the four guiding principles for social innovation that the state just stated. These concepts promote social innovative behaviors in a variety of ways, allowing them to thrive despite a variety of societal issues. In conclusion, the findings of the study are very helpful in reducing social issues for the executives of SOs, government agencies that fund these organizations, and academicians.

The article "Mediating the performance of social organizations in context of social and organizational innovations in China" was retracted in 2024. Reasons: concerns about the data; concerns about the results or conclusions; concerns about the peer review; concerns about the authorship.

## 5. Implications

This study makes an important contribution to scholarly discussion in the perspective of social organizations in developing countries, where there is not only a scarcity of research but also inconclusive results. In context of empirical evidences, this study is a valuable addition for the executives of social organizations; responsible for monitoring and promotion of persons in government entities and similar organizations, donors of resources intended to make a contribution in alleviation of social issues through the intermediation of SOs, the beneficiaries themselves, and generally, for persons who are interested in the issues of SOs.

No doubt, SOs play a significant role in nations to solve social problems of the less privileged segments of the population; however, there is a need for these organizations to become more efficient in accomplishing their goals, as society demands SOs that make the best use of resources from their donors.

The findings are also beneficial for the development and improvement in quality of life in developing economies like China, where there is a huge mobilization of resources for projects of social development and these projects are executed by social organizations of these countries. The positive relationship between performance of social organizations and innovations found by [18], it can be argued that actions of social innovation have a significant impact on organizational performance and these organizations become efficient and effective so geared toward social development.

Organizations can assess their effectiveness using performance measures. This study makes significant contributions in the field of SOs, because their strategy is to participate in development of marginalized communities. As a result, relief delivered through social projects has a stronger impact on a massive population of the country. This demonstrates that these organizations are committed to deliver social services and supporting community development, among other things, and innovations may be a valuable addition in performance of social organizations.

The study has some limitations also. The method used for collection of data is based on non-probabilistic sampling, because it is more user friendly approach so it is biasedness in collecting the information so generalization of results is limited. So future studies may improve this deficiency. In addition, data collection is limited for three provinces of China having higher number of social organizations. Extending the data sample and geographic locations will enhance the scope of the future research.

## Supporting information

S1 Data (XLSX)
